RETRACTED

# Comparison of Efficacy and Psychology of Breast-Conserving Surgery and Modified Radical Mastectomy on Patients with Early Breast Cancer under Graded Nursing

**DOI:** 10.1155/2022/4491573

**Published:** 2022-09-16

**Authors:** Tiantian Ren, Jianli Wu, Lu Qian, Jing Liu, Kan Ni

**Affiliations:** Department of Thyroid and Breast Surgery, Affiliated Hospital of Nantong University, Nantong, Jiangsu 226000, China

## Abstract

**Objective:**

To compare the efficacy and psychology of breast-conserving surgery and modified radical mastectomy in patients with early breast cancer (BC) under graded nursing.

**Methods:**

Forty-one early breast-conserving surgery BC patients admitted to our hospital from April 2020 to March 2022 were regarded as group A, and 52 with modified radical surgery were seen as group B. The operating time, intraoperative bleeding, postoperative drainage, and hospital stay were compared, and the postoperative adverse effects were counted. In addition, patients' psychology and quality of life were assessed using the HAMD, HAMA, and QLSBC rating scales. At the time of discharge, a treatment satisfaction survey was conducted.

**Results:**

The operative time, intraoperative bleeding, postoperative drainage, and hospital stay of patients in group A were lower than those in group B (*P* < 0.05). After treatment, the HAMD and HAMA scores were lower in group A than in group B, while the QLSBC scores and treatment satisfaction were higher (*P* < 0.05).

**Conclusion:**

Breast-conserving surgery under graded nursing is less damaging to early BC patients. It can effectively shorten the postoperative recovery process and improve the psychology and quality of life, so it has higher clinical applicability.

## 1. Introduction

Breast cancer (BC), an extremely common clinical malignancy, has a high incidence worldwide [1]. It mostly occurs in the mammary duct epithelium, and middle-aged and older women are the most prevalent group, and the incidence has shown a younger trend [2]. With the continuous development of modern medical technology, the rate of early BC diagnosis is increasing, and surgical treatment remains the best treatment option. Traditional radical mastectomy requires the entire breast and surrounding tissues to be removed due to the large excision range, which is rarely used in clinical practice [3]. The modified version of radical surgery has gradually developed into a common clinical procedure because of the surgical preservation of the pectoralis muscle and better postoperative appearance [4]. However, for young women, the lack of breasts after radical surgery will greatly impact the patient's self-esteem, affect future marital relationships, breastfeeding, etc., making patients prone to anxiety, depression, low self-esteem, and other negative emotions, affecting the treatment effect [5]. But breast-conserving surgery can effectively solve this problem without affecting the treatment effect, and improve the aesthetics of BC treatment [6].

RETRACTED

In modern health care, the intervention of nursing tools is likewise one of the most vital aspects of improving patient outcome [7]. Several studies have shown the positive impact of applying individualized care strategies for various types of oncology patients [8], but there is still a lack of uniform clinical standard guidelines for BC. Through access to literature, we discovered that graded nursing is a type of service that is graded according to the severity of illness of patients and implemented in a targeted, detailed, and precise manner in relation to their actual condition [9]. It has been shown to exert excellent effects in the surgical treatment of diseases such as gastric cancer and lung cancer [10]. Recently, our hospital has been gradually promoting the use of graded nursing in all departments and expects to improve the quality of medical services and patients' treatment experience in this way.

Thus, this research will provide a reliable reference and guidance for future clinical treatment of early BC patients by comparing the assessment of outcomes and the impact of psychology between breast-conserving surgery and modified radical surgery under graded nursing.

## 2. Materials and Methods

### 2.1. Study Area

The study was carried out at Department of Thyroid and Breast Surgery, Affiliated Hospital of Nantong University from April 2020 to April 2022.

### 2.2. General Data

Ninety-three patients with early BC admitted to our hospital from April 2020 to March 2022 were enrolled to this research. Among them, 41 patients received breast-conserving surgery were regarded as group A, and 52 with modified radical mastectomy were considered as group B. All the above subjects signed the informed consent form.

### 2.3. Inclusion and Exclusion Criteria

Inclusion criteria: all the selected patients were confirmed as early BC by pathological examination, and all of them chose to be treated in our hospital after diagnosis; patients have not received chemotherapy, radiotherapy, or endocrine therapy either preoperatively or prior to puncture; those with TNM stage I-II (The staging standard is based on the BC Staging Guidelines [11]) and those with complete medical records; patients or their immediate family members signed an informed consent form.

Exclusion criteria: those with other malignancies; those with multiple chronic diseases; those with cardiovascular and cerebrovascular diseases; those with organ dysfunction; those with drug allergies; those who suffer from mental illness or physical disability that prevents them from taking care of themselves; contraindication to surgery; transferred patients.

RETRACTED

### 2.4. Hospitalization Management

Both groups of patients were admitted to the hospital using graded nursing [12]. The nursing team was led by the head nurse to establish a nursing plan, standardize the process and quality, and give patients a grade classification based on their own conditions, and implement targeted measures considering the classification. It is more helpful for patients with complex conditions to receive timely and active intervention and ensure the quality of nursing. Furthermore, nurses should help patients prepare for operation, including notification of surgical procedures, presentation of successful cases, and emotional counseling. After surgery, patients' vital signs are closely observed, healthy diet is instructed, upper limb function exercises are carried out in a timely manner, and professional guidance is provided to improve their discomfort and prognosis.

### 2.5. Operation Treatment

The surgeries of both groups were performed by the same surgical team in our hospital. Group A: with the lesion as the center, radial, transverse, or curved incision was chosen according to the location of the tumor, and the base of the tumor and normal breast tissue were excised at 1 cm from the tumor. The excised tissues were subjected to rapid cryopathological examination to mark the internal, external, upper, lower, and basal locations of the incision margin. When the diagnosis is positive at the incision margin, it is necessary to expand the excision again until the test is negative. Then, lymph node dissection is performed in the range of axillary vein, deep surface of pectoralis minor muscle and anterior border of latissimus dorsi muscle, and a drainage tube is disposed in the incision, sutured, and pressure bandaged. Group B: after intravenous compound inhalation anesthesia, the surgical incision was decided according to the size of the affected breast and the location of the tumor, etc. The surgical incision was made 2-5 cm from the outer edge of the tumor and a fusiform incision was made. After cutting the skin of patients' affected breast, the affected breast was excised from the surface of the pectoralis major muscle using an electric knife to free the flap superiorly to the clavicle, inferiorly to the superior edge of the rectus abdominis sheath, internally to the parasternal sternum, and externally to the anterior edge of the latissimus dorsi. Patients' axilla was disposed of by making an incision and lifting the pectoralis major and pectoralis minor muscles inward and upward with a thyroid pull hook to fully expose his axilla. The axillary lymph nodes on the affected side of patients and the lymph nodes between the pectoralis major and minor muscles were removed. Patients' surgical wound was irrigated and soaked using distilled water (45°C), followed by routine placement of a drainage tube and suturing of the incision.

RETRACTED

### 2.6. Outcome Measures

The operative indexes of both groups were compared, including operation time, intraoperative blood loss, postoperative drainage, and hospital stay. The postoperative complications of the two groups of patients were counted, and the incidence of complications = the number of complications/total number × 100%. And the treatment satisfaction before discharge was calculated through the self-made satisfaction scale, the alternative answers are very satisfied, satisfied, dissatisfied, total satisfaction = (very satisfied + satisfied)/total × 100%. The psychological scores after treatment were evaluated by HAMD [13] and HAMA [14] scores, HAMD includes 17 survey items, HAMA includes 14 survey items, and the alternative answers are asymptomatic (0 points), mild (1 point), moderate (2 points), severe (3 points), and very severe (4 points), the higher the score, the more severe the depression and anxiety. The Quality-of-Life Scale for BC (QLSBC) [15] was used to assess the posttreatment quality of life in both groups, including four dimensions of physical functioning, social functioning, psychology, and faith factors, with higher scores indicating higher quality of life.

### 2.7. Statistical Methods

Data were analyzed statistically using SPSS24.0 software. Thereinto, the counting data were represented as (%) and compared through the chi-square test, while the measurement data were expressed in (^−^*χ* ± *s*) and assessed through *t*-test and paired *t*-test. The difference was statistically marked (*P* < 0.05).

## 3. Results

### 3.1. Summary of Results

The operative time, intraoperative bleeding, postoperative drainage, and hospital stay of patients in group A were lower than those in group B (*P* < 0.05). After treatment, the HAMD and HAMA scores were lower in group A than in group B, while the QLSBC scores and treatment satisfaction were higher (*P* < 0.05).

### 3.2. Baseline Data Comparison

The general data such as age and BMI of patients were counted (Table 1). Both groups revealed no statistical difference (*P* > 0.05), suggesting that there was comparability between groups and that subsequent experimental analysis could be performed.

### 3.3. Comparison of Operative Indexes between Groups

It can be seen that the operative time was shorter in group A than in group B (59.07 ± 9.79 min *vs.*96.19 ± 12.85 min, *P* < 0.05, Figure 1(a)). The intraoperative bleeding in group A was (45.95 ± 8.27 mL), also lower than group B (*P* < 0.05, Figure 1(b)). The postoperative drainage was lower in group A than in group B (*P* < 0.05, Figure 1(c)). The length of stay in group A was (3.36 ± 0.88 d), which was dramatically shorter than that in group B (*P* < 0.05, Figure 1(d)).

RETRACTED

### 3.4. Comparison of Postoperative Adverse Reactions

In group A, 2.44% (1 case) of patients had incision infection, 2.44% (1 case) had nausea and vomiting, 2.44% (1 case) had upper limb swelling, and 2.44% (1 case) had subcutaneous effusion. The total incidence of adverse reactions was 9.76%. While in group B, 1.92% (1 case) of patients had incision infection, 3.85% (2 cases) had nausea and vomiting, 3.85% (2 cases) had upper limb swelling, 1.92% (1 case) had flap necrosis, and 1.92% (1 case) had subcutaneous effusion. The total incidence was 13.46%. There was no marked difference in the incidence of postoperative adverse reactions between groups (*P* > 0.05, Table 2).

### 3.5. Comparison of Psychology before and after Treatment

Changes in patients' psychology are equally one of the important aspects that need to be brought to clinical attention in healthcare services nowadays. Thus, we compared the changes in psychological scores of patients before and after treatment. It turned out that the differences in HAMD and HAMA scores before treatment were not statistically obvious (*P* > 0.05). The HAMD score in group A was (8.78 ± 3.18) after treatment, which was lower than that in group B (*P* < 0.05, Figure 2(a)) The HAMA score was (8.34 ± 3.50), which was similarly lower than in group B (*P* < 0.05, Figure 2(b)). In addition, the HAMD and HAMA scores were remarkably lower in both groups after treatment than before treatment (*P* < 0.05).

### 3.6. Comparison of Quality of Life before and after Treatment

Likewise, quality of life, another aspect of modern clinical services that deserves attention, is a direct reflection of patient recovery and prognosis to a large extent. There was no difference in the scores of each dimension of QLSBC score between groups before treatment (*P* > 0.05), while the somatic function score in group A was (58.10 ± 5.64) after treatment, which was dramatically higher than that in group B (*P* < 0.05, Figure 3(a)). But the psychology score in group A was (76.93 ± 4.34), also dramatically higher than in group B (*P* < 0.05, Figure 3(b)). The social functioning domain scores of patients in group A were also higher than those in group B (*P* < 0.05, Figure 3(c)). And the faith factor score in group A was (44.46 ± 5.58), which was higher than that in group B (35.87 ± 7.21), (*P* < 0.05, Figure 3(d)).

RETRACTED

### 3.7. Treatment Satisfaction Comparison

The treatment satisfaction survey in both groups denoted that 58.54% of patients in group A were very satisfied and only 7.32% were dissatisfied, with an overall satisfaction rate of 92.68%. While only 36.54% of patients in group B rated very satisfied, and 26.92% rated unsatisfied, for a total rate of 73.08%. The total satisfaction was dramatically higher in group A than in group B (*P* < 0.05, Table 3).

## 4. Discussion

BC, one of the most common female tumors, has seriously affected the lives of more than 1.2 million female patients worldwide [16]. For early BC, timely surgical procedures can effectively mitigate the pathological development of BC and provide for patient safety [17]. However, because the tumor lesion invades normal breast tissue, most patients may require total removal of the entire breast tissue during surgery [18]. And that is why it is also necessary to pay closer attention to the changes in *x* patients to soothe the psychological burden caused by mastectomy and provide them with prognosis [18]. Graded nursing, one of the common nursing strategies clinically, has achieved extremely excellent results in the treatment of dementia and diabetes [19, 20], but its effectiveness in BC is indistinct.

Currently, personalized care strategies are also one of the extremely important key aspects in modern oncological diseases. Among them, graded nursing, as an excellent nursing management model, has the core concept of patient-centeredness and different treatment measures for patients' conditions through environmental management, psychological guidance, health education, and adjustment of restraint measures under the guidance of nursing humanistic care principles and other methods. It cannot only improve their hospital comfort and eliminate negative emotions but also enhance their treatment effects and recovery to a certain extent [21, 22]. In the case of BC surgery patients, this research can lay the foundation for further promotion and application of subsequent graded nursing. In previous studies, graded nursing has achieved excellent results in the treatment of diabetes, meningioma, and other diseases, and it has been found to improve the nursing efficiency of cardiothoracic surgery patients and alleviate the negative emotions of patients [23–25]. At present, the idea that “individualized nursing strategies can improve the overall recovery of the disease” has been unanimously recognized by the clinic [26]. Therefore, for patients with BC surgery, the application of this study can provide a reliable reference for the follow-up treatment and nursing of BC, further protect the life safety of patients, and lay a foundation for the promotion and application of graded nursing.

RETRACTED

First, we compared the surgical conditions of both groups, and the operative time, intraoperative bleeding, postoperative drainage, and hospital stay of patients in group A were shorter than those in group B, suggesting that our breast-conserving surgery is less damaging to those with early BC and can effectively shorten their postoperative recovery. In a previous study, we also found that the postoperative recovery process was shorter in patients undergoing breast-conserving surgery than those with conventional radical surgery [27], which could also verify the accuracy of this experiment. The feasibility of breast-conserving surgery was confirmed in the NSABP B-06 study in 1995 [28]; because breast-conserving surgery removes only a small area of tissue within the breast when removing the tumor, it can avoid the invasive operation of modified radical surgery with extensive removal of breast contents, skin flaps, and other tissues to a certain extent. So, it causes less damage to the tissues surrounding the lesion within the breast and shortens the postoperative recovery time of patients [29]. Besides, breast-conserving surgery cannot only preserve the breast to the maximum extent and ensure its shape and function to meet the cosmetic needs of patients as much as possible but also safeguard the psychology of patients and reduce the possibility of negative emotions [30]. In the follow-up investigation of the psychology scores of both groups, we also found that the postoperative HAMD and HAMA scores of patients in group A were lower than those of group B, indicating that the postoperative psychology of patients with breast-conserving surgery was more excellent. The lower psychological burden caused by breast-conserving surgery on patients has been mentioned several times in previous studies [31, 32]. In addition, in previous studies, we also found that graded care can also improve the psychological state of stroke and pancreatitis [33, 34], so the improvement of psychological state of patients in the two groups may also be affected by graded care. But this effect is positive for the patient's recovery. Nevertheless, we found no statistical difference in the incidence of adverse reactions between groups, which may be due to statistical contingency caused by small number of cases. It may also be because the subjects were all early BC patients, and therefore generally had a better postoperative recovery and a lower incidence of adverse effects. This will be verified as soon as possible in the follow-up experiments. Finally, we compared the quality of life between both groups, and the QLSBC score of patients in group A was higher, which indicated that the quality of life of those undergoing breast-conserving surgery was better after treatment. And this we presume is also because breast-conserving surgery causes less damage to patients. Meanwhile, the improvement of patients' negative emotions can more effectively enhance their postoperative recovery and quality of life. More than that, the treatment satisfaction rate was also higher in group A than in group B. It also once again indicates that breast-conserving surgery is more applicable in BC treatment and more recommended for clinical preference. Of course, the application of breast conserving surgery in the treatment of BC has been clinically verified many times [35, 36], and this study further highlights the future significance of breast conserving surgery in the treatment of BC through the comparison with modified radical mastectomy. This will undoubtedly be of great help to the choice of surgical treatment for BC patients.

RETRACTED

## 5. Conclusion

Breast-conserving surgery under graded nursing is less damaging to early BC patients. It can effectively shorten the postoperative recovery process and improve the psychology and quality of life, so it has higher clinical applicability.

## Figures and Tables

**Figure 1:** Comparison of surgical indicators between groups. (a) Comparison of operative time between groups. (b) Comparison of intraoperative bleeding between groups. (c) Comparison of postoperative drainage between groups. (d) Comparison of length of stay between groups. ^∗∗∗^*P* < 0.005.

**Figure 2:** Comparison of psychology before and after treatment. (a) Comparison of HAMD scores of both groups before and after treatment. (b) Comparison of HAMA scores of both groups before and after treatment. ^∗∗∗^*P* < 0.005.

**Figure 3:** Comparison of quality of life before and after treatment. (a) Comparison of somatic function scores of both groups before and after treatment. (b) Comparison of psychology scores of both groups before and after treatment. (c) Comparison of functioning domain scores of both groups before and after treatment. (d) Comparison of faith factor scores of both groups before and after treatment. ^∗∗∗^*P* < 0.005.

**Table 1:** Baseline datasheet.

	Group A (*n* = 41)	Group B (*n* = 52)	*t* or *χ*^2^	*P*
Age	64.07 ± 4.95	62.77 ± 9.27	0.811	0.420
BMI (kg/m2)	26.11 ± 3.03	25.32 ± 3.33	1.181	0.241
Living environment			0.862	0.353
In the city	26 (63.41)	28 (53.85)		
In the countryside	15 (36.59)	24 (46.15)		
Type of cancer			0.797	0.372
Ductal cancer	41 (100.0)	51 (98.08)		
Lobular cancer	0 (0.0)	1 (1.92)		
Drinking			0.001	0.982
Yes	4 (9.76)	5 (9.62)		
No	37 (90.24)	47 (90.38)		
Family history of illness			0.145	0.703
Have	1 (2.44)	2 (3.85)		
None	40 (97.56)	50 (96.15)		
Pathological stage			0.091	0.764
Stage I	21 (51.22)	25 (48.08)		
Stage II	20 (48.78)	27 (51.92)		

RETRACTED

**Table 2:** Postoperative adverse reactions.

	Incision infection	Nausea and vomiting	Upper limb swelling	Flap necrosis	Subcutaneous effusion	Total incidence (%)
Group A (*n* = 41)	1 (2.44)	1 (2.44)	1 (2.44)	0 (0.00)	1 (2.44)	9.76
Group B (*n* = 52)	1 (1.92)	2 (3.85)	2 (3.85)	1 (1.92)	1 (1.92)	13.46%
*χ* ^2^						0.302
*P*						0.583

**Table 3:** Treatment satisfaction survey.

	Very satisfied	Satisfied	Dissatisfied	Total satisfaction (%)
Group A (*n* = 41)	24 (58.54)	14 (34.15)	3 (7.32)	92.68
Group B (*n* = 52)	19 (36.54)	19 (36.54)	14 (26.92)	73.08
*χ* ^2^				5.899
*P*				0.015

## Data Availability

The datasets used and/or analyzed during the current study are available from the corresponding author on reasonable request.
